The article "A review on microalgae cultivation and harvesting, and their biomass extraction processing using ionic liquids" was retracted in 2026. Reason: compromised peer review.

# A review on microalgae cultivation and harvesting, and their biomass extraction processing using ionic liquids

**DOI:** 10.1080/21655979.2020.1711626

**Published:** 2020-01-24

**Authors:** Jia Sen Tan, Sze Ying Lee, Kit Wayne Chew, Man Kee Lam, Jun Wei Lim, Shih-Hsin Ho, Pau Loke Show

**Affiliations:** a Department of Chemical and Environmental Engineering, Faculty of Science and Engineering, University of Nottingham Malaysia, Semenyih, Malaysia; b Department of Biotechnology, Faculty of Applied Science, UCSI University, Kuala Lumpur, Malaysia; c Department of Chemical Engineering, Lee Kong Chian Faculty of Engineering and Science, Universiti Tunku Abdul Rahman, Sungai Long Campus, Kajang, Malaysia; d School of Mathematical Sciences, Faculty of Science and Engineering, University of Nottingham Malaysia, Selangor, Malaysia; e Chemical Engineering Department, Universiti Teknologi PETRONAS, Perak, Malaysia; f Centre for Biofuel and Biochemical Research, Institute of Self-Sustainable Building, Universiti Teknologi PETRONAS, Seri Iskandar, Malaysia; g Fundamental and Applied Sciences Department, Universiti Teknologi PETRONAS, Seri Iskandar, Malaysia; h State Key Laboratory of Urban Water Resource and Environment, School of Environment, Harbin Institute of Technology, Harbin, China

**Keywords:** Microalgae, cultivation, harvesting, extraction, ionic liquids, downstream processing

## Abstract

The richness of high-value bio-compounds derived from microalgae has made microalgae a promising and sustainable source of useful product. The present work starts with a review on the usage of open pond and photobioreactor in culturing various microalgae strains, followed by an in-depth evaluation on the common harvesting techniques used to collect microalgae from culture medium. The harvesting methods discussed include filtration, centrifugation, flocculation, and flotation. Additionally, the advanced extraction technologies using ionic liquids as extractive solvents applied to extract high-value bio-compounds such as lipids, carbohydrates, proteins, and other bioactive compounds from microalgae biomass are summarized and discussed. However, more work needs to be done to fully utilize the potential of microalgae biomass for the application in large-scale production of biofuels, food additives, and nutritive supplements.

## Introduction

Algae are a group of photosynthetic autotrophs which normally thrives in various types of water bodies such as lakes, rivers, and sea. They are accounted for producing atmospheric oxygen via photosynthesis, which is a process that converts water and carbon dioxide into carbohydrate using solar energy. Algae group is diverse and encompasses numerous different phyla with their own unique characteristics and properties ranging from prokaryotic single cellular cyanobacteria to more complex multicellular eukaryotic algae, as summarized in Table 1.

The article "A review on microalgae cultivation and harvesting, and their biomass extraction processing using ionic liquids" was retracted in 2026. Reason: compromised peer review.

**Table 1.** Classes of algae and their respective characteristics and examples.

Type of algae	Characteristic	Example
Cyanobacteria	Cyanobacteria or blue-green algae are gram-negative bacteria which can survive at some of the harshest habitats on earth. Some of them are known to be able to do nitrogen fixation along with carbon fixation both of which are essential for life on earth.	*Prochlorococcus, Spirulina, Nostoc, Cyanothece, Anabaena*
Glaucocystophytes	Glaucocytophytes are relatively uncommon unicellular eukaryotic algae that contain plastid which is structurally similar to cyanobacteria. Glaucocystophytes are one of the descendants of the product of early endosymbiosis.	*Cyanophora*, *Glaucocystis, Peliaina, Gloeochaete*
Rhodophytes	Rhodophytes or red algae are comprised of mostly multicellular photosynthetic eukaryotes. They are characterized by their distinctive red color due to the presence of red pigments such as phycobilisomes in their chloroplast.	*Batrachospermum, Chroodactylon, Bangia, Cyanidium, Compsopogon*
Chlorophytes	Chlorophytes or green algae are photosynthetic eukaryotes which contain chlorophylls as their main photosynthetic pigments.	*Haematococcus, Chlorella, Dunaliella, Graesiella, Scenedesmus*
Charophytes	Charophytes are mainly terrestrial and freshwater algae. They are notably having similar features as terrestrial plants, suggesting that the ancestors of charophytes gave rise to land plants.	*Coleochaete, Micrasterias, Chara, Penium, Klebsormidium*
Chlorarachinophytes	Chlorarachinophytes are marine photosynthetic protists which possess secondary plastids originated from secondary endosymbiosis.	*Chlorarachnion, Lotharella, Bigelowella*
Euglenoids	Euglenoids are unicellular flagellated eukaryotes which exhibit both animal- and plant-like characteristics. Most Euglenoids are freshwater species while some are marine species.	*Euglena, Discoplastis, Phacus, Colacium, Strombomonas*
Apicomplexans	Apicomplexans are a group of obligate intracellular parasites with which are responsible for causing various diseases in animals and human.	*Plasmodium, Toxoplasma, Cryptosporidium*
Dinoflagellates	Dinoflagellates are a class of unicellular protists and are characterized by their relatively large nuclei, golden-brown-colored plastid and its unique method of swimming.	*Gymnodinium, Karenia, Dinophysis, Alexandrium*
Heterokontophytes	Heterokontophytes are flagellated photosynthetic eukaryotes. They are characterized by their biflagellate which is different in length.	*Chrysophyacae, Parmophyaceae, Xanthophyacae, Dictyophyaceae*
Haptophytes	Haptophytes are unicellular photosynthetic microalgae with its chloroplast originated from the endosymbiosis of red algae. It usually has 2 equal or unequal flagella which allow it to be motile.	*Chrysochromulina, Prymnesium, Pavlova, Diacronema*
Cryptophytes	Cryptophytes are motile, and photosynthetic unicellular organisms characterized by the presence of 2 flagella and are typically found in freshwater and marine habitat.	*Guillardia, Campylomonas, Geminigera, Rhodomonas, Teleaulax*

Under the group of algae, microalgae are unicellular microorganisms which thrive in both saltwater and freshwater environments. Despite the absence of complex structure and organs when compared to their plant cousins, microalgae are able to perform photosynthesis using sunlight, carbon dioxide and water owing to the presence of photosynthetic pigments such as chlorophylls in their cells. Microalgae species have provided a limitless opportunity for being utilized in different sectors for the benefits of mankind [1]. Human has cultivated microalgae such as *Spirulina* for their nutritive properties [2]. Besides, microalgae contain various valuable bioactive compounds which can be derived from their cells, including lipids, proteins, carbohydrates, carotenoids, and vitamins. These valuable bioactive compounds can be widely used in commercial applications.

The article "A review on microalgae cultivation and harvesting, and their biomass extraction processing using ionic liquids" was retracted in 2026. Reason: compromised peer review.

However, many microalgae species still remain underutilized and numerous researchers have explored many different possibilities to fully utilize microalgae. Ionic liquids (ILs) have emerged among other candidates which appreciate the vast amount of precious bio-compounds that reside within microalgae. The tunable solvent properties of ILs enable them to extract a wide range of bio-compounds from microalgae biomass at a comparative raw material and energy utilization compared to the conventional method available. Therefore, besides evaluating the technologies being studied recently for microalgae cultivation and harvesting, this review focuses on the extraction of bio-compounds from microalgae using ILs as extractive solvents. To be more specific, the use of ILs as extractive solvents using different techniques such as microwave-assisted IL extraction, ultrasound-assisted IL extraction, and IL-based aqueous biphasic systems (ABS) are discussed, and the recent works are summarized.

## Microalgae cultivation

Microalgae are capable to grow rapidly. Their high photosynthesis efficiency coupled with the ability to accumulate a large amount of bioproducts within their cells make them a suitable candidate to serve as industrial raw material [1]. Besides, cultivation of microalgae does not require fertile land, a large quantity of freshwater, and herbicides and pesticide when compared to the other crops and thus will not be competing for resources [3]. Furthermore, cultivation of microalgae can even be performed using wastewater such as domestic sewage water and palm oil milling effluents which can assist in bioremediation of wastewater [4,5]. Apart from wastewater treatment, cultivation of microalgae can also help with reduction of atmospheric carbon dioxide through photosynthesis, effectively contributing to the efforts of tackling greenhouse effect and global warming. Despite the benefits of microalgae cultivation, its developments are still plagued with various problems. For example, the low biomass production and the small size of cells when they are cultured in liquid medium render the harvesting process of microalgae very costly.

The article "A review on microalgae cultivation and harvesting, and their biomass extraction processing using ionic liquids" was retracted in 2026. Reason: compromised peer review.

One of the ways to work around the shortcomings of usage of microalgae in the industry is by increasing their growth rate to compensate for their low cell density and difficulties in harvesting. Numerous equipment and technologies have been improved across the years to ramp up the production of microalgae. Although microalgae can be easily cultured in a highly controlled laboratory condition, however, it is still harder to ensure the high productivity of microalgae in large-scale production. An ideal microalgae culturing system should possess the characteristics, including: (1) adequate light source, (2) effective transfer of material across liquid-gas barrier, (3) simple operation procedure, (4) minimal contamination rate, (5) cheap overall building and production cost, and (6) high land efficiency [6]. In general, microalgae culturing system can be broadly classified into two categories, which are the open pond and photobioreactor. Each system has its pros and cons.

### Open pond

Open pond cultivation has been one of the oldest and simplest ways to cultivate microalgae in large scale. Open pond is widely used in the industry due to its relatively cheaper construction, maintenance and operation cost. Other advantages of using open pond system include simplistic operation and maintenance, low energy demand, and ease to scale up [7]. There are few types of open pond, which includes natural water such as lakes and ponds, and artificial water bodies such as circular and raceway ponds. At some cases, a container such as a tank can also be used to culture microalgae [8]. Open pond system has the advantage of being the most cost-efficient cultivation system. However, despite the large cultivation area, cultivation of microalgae from natural water has relatively lower cell concentration and thus a highly efficient harvesting method is required [9]. In addition, issues such as rainwater runoff which affects the growth condition of microalgae such as salinity and pH, erosion of banks that resulting in leakage and increased water turbidity might significantly affect the productivity of microalgae in open ponds [10]. Another issue that presents in open pond cultivation system is the possibility of contamination by protozoa and bacteria which causes the products to be toxic and unusable. The current available way to circumcise this problem is by cultivating microalgae which are capable of surviving at extreme alkaline or saline condition since only a few contaminants are able to thrive under this condition [11,12]. Besides, due to the open nature of the system, it is harder to control certain growth parameters such as temperature and light intensity which might affect the growth rate of microalgae [11].

The article "A review on microalgae cultivation and harvesting, and their biomass extraction processing using ionic liquids" was retracted in 2026. Reason: compromised peer review.

Harvesting of microalgae from naturally occurring sources has been one of the oldest microalgae cultivation techniques known to man. The oldest record of microalgae harvesting was done by Aztec peoples where they harvest *Spirulina* from Lake Texcoco located at Mexico [13]. This cultivation method highly depends on naturally occurring water bodies to provide right condition and nutrients for the growth of microalgae. Currently, one of the largest commercial cultivation of microalgae in natural water is located at Hutt Lagoon, Australia which is capable of producing 6 tons of β-carotene every year form *Dunaliella* using its 700-hectare ponds [10].

Circular ponds are the first artificial pond to be used in large-scale cultivation of microalgae. This cultivation system got its name from its circular-shaped culture tank, and typically have the depth of 30–70 cm and width of 45 m along with a rotating agitator located at the center of the pond [14]. The rotating agitator is being used to ensure efficient mixing and prevent sedimentation of algae biomass [15]. However, the design of this cultivation system is limited by its size since bigger pond might introduce stronger water resistance, and therefore causes strain on the mechanical parts of agitator [16]. Moreover, this design has disadvantages for high energy usage in the agitation process and high construction cost [13]. Currently, this cultivation system has been used in Japan and Taiwan to culture *Chlorella* for consumption [14,17].

Raceway pond is one of the most frequently used open pond types for the cultivation of microalgae. It consists of a series of closed loop channel around 30-cm deep and paddlewheel which enable recirculation of microalgae biomass to ensure equal distribution of nutrients and prevent sedimentation of microalgae biomass. Raceway pond has been perceived as one of the best open pond cultivation design available due to its energy efficiency, as a single paddlewheel is sufficient enough to properly agitate a 5-hectare raceway pond [18]. One of the successful raceway pond cultivation is by Sapphire Energy’s Columbus Algal Biomass Farm located at Columbus, United States, which has successfully produced 520 metric tonnes of dried microalgae biomass during 2 years of its operation without any technical issue [19].

The article "A review on microalgae cultivation and harvesting, and their biomass extraction processing using ionic liquids" was retracted in 2026. Reason: compromised peer review.

### Photobioreactor

Photobioreactor is a bioreactor system used to culture phototrophs such as microalgae in an enclosed system which does not allow direct exchange of material between the culture and environment. Photobioreactor is able to overcome several constraints faced commonly by open pond culture design. First, the size of bioreactor is more compact compared to open pond, therefore providing more efficient land usage. Second, the system provides a closed and highly controlled growth condition for the culture, thus able to produce a contamination free, single strain microalgae culture [20]. In addition, the highly controlled culture condition can also translate into higher nutrient and metabolic efficiency which results in higher biomass production per unit of substrate. However, the bottleneck of practical usage of photobioreactor is its limited scalability due to various design flaws, rendering it uneconomical to be used in large-scale production [21]. Moreover, highly controlled growth condition of photobioreactor always comes with high capital and operating costs.

Tubular photobioreactor is comprised of transparent long tubes made out of glass or transparent plastics which are arranged in horizontal, vertical, helix, or slanted orientation to maximize capture of sunlight [13,22]. The microalgae culture is circulated within the loop by the means of mechanical pump or air lift system [23]. However, the biggest drawback of tubular photobioreactor design is in its poor mass transfer across the system since the long tube used in the bioreactor design might result in the differences in concentration of substrate and product along the tubes. Commercial usage of large-scale tubular photobioreactor is being used to produce *Haematococcus* and *Chlorella* at Germany and Israel, respectively [24].

Vertical column bioreactor is constructed by a transparent vertical cylindrical tubing and a sparger which pumps in air bubbles to enable homogenization of the culture and allow transfer of carbon dioxide and oxygen between air and microalgae culture [25]. This culture system offers the best gas-liquid mass transfer efficiency compared to other system owing to the capability of the sparger used in this system to generate smaller bubbles which provide larger total surface area for more efficient transfer of substance [26]. In addition, the simplicity of the design allows it to have lower energy demand and simpler operating procedure. However, the cylindrical-shaped container does not provide adequate amount of light required by the microalgae to perform photosynthesis efficiently. Moreover, high construction cost and difficulties in cleaning the reactor make commercial usage of vertical column photobioreactor difficult [27]. Commercial usage of this photobioreactor design has yet to be found, however, numerous large-scale experimental reactor has been made including a 40-liter vertical column outdoor photobioreactor for the cultivation of *Chlorella zofingiensis* at Guangdong, China [28].

The article "A review on microalgae cultivation and harvesting, and their biomass extraction processing using ionic liquids" was retracted in 2026. Reason: compromised peer review.

Flat-plate photobioreactor on the other hand is characterized by its rectangular-shaped compartment made out of transparent material with the depth between 1 and 5 cm. The culture inside the reactor is mixed via the means of recirculating airlift system [29]. This design supports the largest total surface area for illumination and low oxygen build up, thus achieving the highest photosynthetic efficiency out of all photobioreactor design [30]. However, the aeration design of this photobioreactor causes stress damage to the microalgae cells [31]. Numerous innovative design has been implemented to further improve the efficiency of the flat-plate photobioreactor, such as twin layer flat-plate and plastic sheets photobioreactors [32]. Commercial usage of flat-plate photobioreactor has been used to produce astaxanthin by Algamo company located at Krkonoše, Czech Republic.

## Harvesting of microalgae

Harvesting of microalgae is one of the main parts in microalgae processing. Several studies have suggested that it makes up 20–30% of the total production cost due to high energy demand and capital cost [33,34]. In general, all harvesting techniques aim to remove as much culture media from the microalgae biomass to facilitate next downstream processing such as extraction of bioactive compounds. Numerous harvesting methods have been used to collect biomass, including filtration, centrifugation, flocculation, and flotation [35]. For some circumstances, a combination of two or more techniques are employed to further increase harvesting efficiency. Table 2 presents several harvesting approaches and their respective target microalgae species, advantages, and disadvantages.

**Table 2.** Various harvesting methods, and their respective target microalgae species and advantages.

Harvesting technique	Microalgae species	Advantage	Disadvantage	Reference
Cross flow filtration	*Chlorella* sp.	High energy efficiency	Prone to membrane fouling and shearing of fragile materials	[36]
Axial vibration membrane filtration	*Chlorella pyrenoidosa*	Reduced membrane fouling	Require power-consuming pumping units	[37]
Polyacrylonitrile-based membrane filtration	*Scenedesmus* and *Phaeodactylum*	Reduced membrane fouling	Require power-consuming pumping units	[38]
Tilted membrane panel filtration	Wild microalgae strain	Reduction of membrane cost, and energy consumption	Membrane fouling	[39]
Ultrafiltration	*Dunaliella salina*	Less cell shearing, low energy and chemical consumption	High capital cost	[40]
Electro-flocculation	*D. salina*	Cost efficient and chemical free	High energy demand	[41]
Plant bio-flocculation (*Moringa oleifera*)	*Chlorella* sp.	Cost efficient and limited toxicity	Contamination of microalgae products	[42]
Microbial bio-flocculation	*Desmodesmus brasiliensis*	Cost efficient and biodegradable	Contamination of microalgae products	[43]
Chemical flocculation	*Chlorella* sp.	Cost efficient and ease for up scale	Utilization of toxic chemicals	[44]
Buoy-bead flotation	*Chlorella vulgaris*	Chemical free and high reusability	High cost	[45]
Magnesium coagulation-dissolved air flotation	*Chlorella zofingiensis*	Does not utilize external coagulant and high recyclability of coagulant and biomass	Utilization of toxic chemicals	[46]
Electrolytic flotation	*C. vulgaris*	Chemical free, low energy demand and can be used in continuous system	High operating and capital cost	[47]
Foam flotation	*C. vulgaris, Isochrysis galbana*, and *Tetraselmis suecica*	Low cost and energy demand, highly scalable	High operating and capital cost	[48]
Ozone flotation	*Scenedesmus* sp.	Increased microalgae bio-compound recovery	Require specialized ozone generation equipment onsite	[49]

The article "A review on microalgae cultivation and harvesting, and their biomass extraction processing using ionic liquids" was retracted in 2026. Reason: compromised peer review.

### Filtration

Filtration process utilizes a semipermeable membrane which can retain microalgae on the membrane while allowing the liquid media to pass through, leaving the algae biomass behind to be collected [50]. This method can harvest high concentration of cell from the medium, and the varying pore size of the filter membrane enables the system to suit the need of different microalgae and are able to handle the more delicate species which are prone to damage due to shearing. However, this method is very prone to fouling and clogging and therefore requires frequent change of fresh filter or membrane that might contribute significantly to its processing cost [51]. In view of this constraint, filter membrane using cheap and easily accessible material has been developed. Bejor and his colleagues [52] have successfully developed a filter membrane made out of stretch cotton which can achieve harvesting efficiency of 66–93%.

### Centrifugation

Centrifugation operation separates microalgae cells from the culture media based on each component’s density and particle size using centrifugal force [53]. This technique has high cell harvesting efficiency, but the process is time consuming and energy intensive [54,55]. Moreover, high gravitational force used in centrifugation might cause cellular damage making it unfavorable for certain applications since the sensitive nutrients might be lost [56,57]. Several types of centrifugal systems have been used in the industry; these include disk stack centrifuges, perforated basket centrifuges, imperforated basket centrifuges, decanters, and hydro-cyclones [35].

### Flocculation

Flocculation is a process where free floating unicellular microalgae cells aggregate together to form a larger particle known as floc by the addition of flocculating agent to remove the surface charge of cells [58]. Flocculating agents can be grouped into two major types, namely chemical flocculants and bio-flocculants. Low cost and highly available chemical flocculants such as iron and aluminum salts have been used widely in industry [59]. The study carried out by Chatsungnoen and Chistt [60] has demonstrated that the metal salts such as aluminum sulfate and iron chloride are able to remove 95% of the microalgae biomass at a standard condition. However, the chemicals are not eco-friendly due to their high toxicity, and they must be removed by additional treatment processes which add to the production cost [61].

Bio-flocculants on the other hand are much safer and eco-friendly when compared to their chemical counter parts. They are also cheaper to be used, and typically there is no pretreatment required before further downstream processing of microalgae and recycling of culture media [62,63]. Most of the bio-flocculants used are biopolymers such as acrylic acid and chitosan which exist naturally or produce artificially [64]. It is reported that chitosan at a lower dosage is capable of reaching 90% cell recovery when compared to chemical flocculants such as aluminum sulfate which requires higher concentration to achieve same results [65].

### Flotation

Flotation utilizes small bubbles which attach on microalgae cells to promote the floating of cells on the surface of the culture media for easy harvesting [66]. The advantages associated with the flotation system include relatively high harvesting efficiency, easy operating procedure, and high processing throughput at low cost [67].

The article "A review on microalgae cultivation and harvesting, and their biomass extraction processing using ionic liquids" was retracted in 2026. Reason: compromised peer review.

There are 3 main types of flotation systems which generate air bubbles required by using different mechanisms. Dissolved air flotation system generates air bubbles by the means of saturating the culture with compressed air and then discharging the culture at atmospheric condition. This method has been widely used in wastewater treatment but is hindered by high cost due to power consumption and usage of chemicals [68]. Dispersed air flotation on the other hand uses a sparger to generate air bubble which in turn have lower energy demand when compared to dissolved air flotation [69]. The third method is electro-flotation, which applies electrolysis operation to generate microbubbles from its electrode to trap free floating microalgae [70]. Apart from harvesting, this method also allows simultaneous cell disruption operation when alternating current is being used [71]. However, the respective system is extremely energy consuming and frequent replacement of electrode is required due to fouling which might then bring up the production cost [35].

## Extraction of bioproducts from microalgae using ionic liquids

Microalgae are known to contain vast amount of high-value phytochemicals. However, since most of the compounds are locked within the rigid cell walls, the extraction of bioactive compounds from microalgae involves cellular disruption to release the intracellular contents so that it could be accessed and purified. Numerous ways have been devised to extract the bioactive compounds from microalgae biomass. Typical conventional extraction method can be broadly classified into four groups which are: (1) mechanical extraction which utilizes shear forces, electrical pulses, waves or heat to disrupt cellular structure [72], (2) chemical extraction which uses different kinds of solvents such as polar or nonpolar organic solvents, supercritical carbon dioxide and ILs to extract the intracellular compounds [73], (3) physical extraction which applies the microwave and ultrasound operations [74], and last (4) enzymatic lysis which employs enzymes such as trypsin to digest the hard cell wall of microalgae [75]. Among all the extraction methods, ILs have emerged as a promising green solvent for the extraction of microalgae bio-compounds, and different approaches using ILs have been examined.

### Ionic liquids as extractive solvents using different approaches

ILs are described as molten organic salts which has melting point below 100℃ [76,77]. The properties of ILs vary greatly depending on their molecular size, functional groups attached, and also the type of cation and anion pairs. Nevertheless, several common characteristics have made IL as an ideal candidate for green applications. First, the nonvolatile nature makes ILs ideal when compared to other organic solvents such as ethanol and methanol which are extremely combustible. Second, some ILs have low viscosity which is a plus for any IL that is intended to be used for large-scale industrial application since low fluid viscosity facilitates pumping and agitation operations and reduce the power consumption [78]. Additionally, the low vapor pressure of ILs makes them relatively safe to use especially when they have low emission rate and consequently reduce exposure toward operators. The negligible vapor pressure of ILs also translate into less air pollution since there is lesser ILs will be liberated into the atmosphere. Furthermore, ILs can be specifically tailored-made to suit specific conditions and to solubilize specific compounds by altering their functional groups or selection of appropriate cation and anion combinations. Moreover, ILs have high thermal and chemical stability, high conductivity, and remarkable solubilizing capacity for various organic and inorganic compounds [79,80].

The article "A review on microalgae cultivation and harvesting, and their biomass extraction processing using ionic liquids" was retracted in 2026. Reason: compromised peer review.

Amongst the commercially available ILs, ILs from imidazolium cation family are widely investigated for their potential to extract bioproducts from microalgae. Imidazolium cation has 5 membered, heterocyclic structure with a pair of nitrogen at the 1st and 3rd position in the ring [81]. Its peculiar structure allows it to be used for various applications. Apart from imidazolium-based ILs, cholinium-based ILs that are highly recognized for their marginally toxicity have been applied for the microalgae extraction studies [82]. However, there is still lack of study in this field using other ILs such as pyridinium- and phosphonium-based ILs.

Several extraction methods using ILs have been studied. Although direct dissolution of microalgae biomass to extract their intracellular compounds is within the realm of possibility, most of the time additional external force is used to aid the extraction process [83]. Microwave, ultrasound, electrical pulse field, and bead milling can be coupled with the use of ILs to generate additional force to intensify the extraction process. These methods are mainly developed to work around the tough cell wall of microalgae that is being a hindrance to the full utilization of microalgae-derived compounds.

#### Microwave-assisted ionic liquid extraction

Microwave employs high-frequency waves to cause vibration of water molecule within the microalgae biomass, which in turn increase the temperature and pressure generated from the evaporation of water resulting in the rupture of cell wall [74,84]. The ruptured microalgae cell releases all its intracellular contents and these contents are freely available to be extracted using ILs. Recent work conducted by Wahidin et al. [85] reported that by using 1-ethyl-3-methylimmidazolium methyl sulfate as extractive solvent and combined with microwave heating, it is possible to convert directly *Nannochloropsis* sp. biomass to biodiesel in a single step *in situ* transesterification process. The approach has achieved efficient biodiesel production per unit of microalgae biomass [85].

The article "A review on microalgae cultivation and harvesting, and their biomass extraction processing using ionic liquids" was retracted in 2026. Reason: compromised peer review.

#### Ultrasound-assisted ionic liquid extraction

Ultrasound induces formation of cavity within microalgae cells, and when the cavity collapses it generates large amount of force which causes the shearing of microalgae cell wall [86]. This method has a high potential for microalgae biodiesel production since it is able to achieve cell disruption without the energy intensive dewatering procedure [87]. Ultrasonic treatment of 25kHz on *Spirulina platensis* suspended in 1:1 ratio ILs mixture of 2-hydroxyethylammonium acetate and 2-hydroxyethylammonium formate has been studied, and experimental results demonstrated that the ILs mixture solution has higher extraction efficiency of phycocyanin, allophycocyanin, and phycoerythrin when compared to conventional sodium phosphate buffer and 1-butyl-3-methylimidazolium chloride [88].

#### Ionic liquid-based aqueous biphasic systems

Beside of being applied in microwave- and ultrasound-assisted ILs extraction, ILs are studied as phase-forming components in ABS for the separation of bioproducts derived from microalgae biomass. ABS can be formed by mixing two different water-soluble ILs which are not immiscible with each other [89,90]. The bioproducts from microalgae can be separated into different aqueous phases based on their physical properties and chemical affinity. It is reported that the ABS formed by 1-butyl-3-methylimidazolium dibutylphosphate and tributylmethylphosphonium methyl sulfate was able to extract protein, fatty acid and carbohydrate from *Neochloris oleoabundans* at 80%, 68%, and 77%, respectively. This low energy demanding method has shown better yield compared to their organic solvent counterparts [91].

### Bioproducts derived from microalgae using ionic liquid technology

Microalgae-derived bioproducts can be categorized into four major groups, namely lipids, carbohydrates, proteins, and bioactive compounds. Table 3 summarizes the recent studies utilizing ILs to extract these bioproducts from microalgae.

**Table 3.** Extraction studies of bioproducts from microalgae using ILs as extractive solvents.

Bioproduct	Microalgae species	IL	Reference
Lipid	*N. oleoabundans*	1-butyl-3-methylimidazolium methyl sulfate	[87]
Lipid	*N. oculata*	Tetrakis(hydroxymethyl)phosphonium chloride	[92]
Lipid	*Chlorella, Chlorococcum* sp. and *Nannochloropsis oculata*	Butyrolactam hexanoate	[93,94]
Lipid	*C. vulgaris*	1-butyl-3-methylimidazolium trifluoromethanesulfonate	[104]
Lipid	*Chlorella sorokiniana, Nannochloropsis salina* and *Galdieria sulphuraria*	1-butyl-3-methylimidazolium hydrogen sulfate	[95]
Lipid	*C. vulgaris*	1-ethyl-3-methyl imidazolium ethyl sulfate, 1-ethyl-3-methyl imidazolium thiocyanate, 1-ethyl-3-methyl imidazolium hydrogen sulfate,	[96]
Fatty acid methyl ester	*C. vulgaris*	1-ethyl-3-methylimidazolium ethylsulfate	[97]
DHA	*Thraustochytrium* sp.	1-ethyl-3-methylimidazolium ethylsulfate, tetrabutylphosphonium propionate	[106]
DHA	*Aurantiochytrium* sp.	Iron(III) chloride hexahydrate, 1-Ethyl-3-methylimidazolium acetate mixture	[98]
Carbohydrate and lipid	*C. vulgaris* and *S. platensis*	Choline L-argininate	[111]
Glucan, arabinan and protein	*I. galbana*	1-methyl-3- octylimidazolium chloride	[99]
Protein	*C. vulgaris*	Cholinium 2-hydroxy-3- morpholinopropanesulfonate	[86]
C-phycocyanin	*S. platensis*	1-octyl-3-methylimidazolium bromide	[100]
Astaxanthin	*H. pluvialis*	1-ethyl-3-methylimidazolium di-butylphosphate	[118]

The article "A review on microalgae cultivation and harvesting, and their biomass extraction processing using ionic liquids" was retracted in 2026. Reason: compromised peer review.

#### Lipids

Microalgae have been known for their richness in lipid content, where the lipid content of the dried microalgae biomass is around 20–50%, however with specific optimized culturing technique the lipid content of microalgae can be risen to 80% [101]. In general, there are two major applications for microalgae-derived lipids, which are biodiesel and food supplement. Microalgae biodiesel is considered as the green fuel for the future owing to its carbon neutrality and the utilization of feedstock which does not compete with our current food supply for resources [101–103]. Several published works have conceptualized the use of ILs to extract lipid from microalgae for biodiesel production. In a study conducted by Zhou and his colleagues [87], 1-butyl-3-methylimidazolium methyl sulfate was able to extract the total lipid of 16.04% from dried *N. oleoabundans* biomass when the ratio of IL: methanol used was 1:1. The extraction efficiency can be further increased to beyond 20% when the IL: methanol mixture utilized was at the ratio of 1:3 and 1:7 under the optimized extraction condition.

*C. vulgaris* is one of the most studied microalgae strains available for biodiesel production. It was reported that 1-butyl-3-methylimidazolium trifluoromethanesulfonate achieved lipid extraction efficiencies of 12.5% and 19% for commercial and cultivated dried *C. vulgaris* biomass, respectively, which were much higher when compared to conventional Bligh and Dyer’s method with extraction efficiency achieved at 10.6% and 11.1% [104,105]. In addition to that, the fatty acid profile of the crude lipid extract from ILs extraction showed that it was rich in palmitic, linoleic, and palmitoleic fatty acids which can undergo a cheap and fast transesterification process with the presence of an acid or alkaline catalysis to produce biodiesel [104]. On the other hand, lipids extracted from microalgae can also be used as food additives to supply additional nutritive factors in human food. The study on the extraction of DHA from *Thraustochytrium* sp. biomass reported 1-ethyl-3-methylimidazolium ethylsulfate and tetrabutylphosphonium propionate, with the use of IL:methanol at 1:10 and 1:4 ratio, respectively, achieved lipid extraction yield of 91% [106].

The article "A review on microalgae cultivation and harvesting, and their biomass extraction processing using ionic liquids" was retracted in 2026. Reason: compromised peer review.

#### Carbohydrates

Microalgae cells are packed with different complex carbohydrates such as cellulose, agarose, starch, and glycogen which can be readily used as feedstock to produce bioethanol [3]. Bioethanol produced from microalgae carbohydrates can be used directly by currently available internal combustion engine without significant modification. In addition, high octane rating and oxygen content of bioethanol fuel translate well into higher engine performance and reduced emission rate [107]. ILs are suitable solvents to extract carbohydrate from microalgae since the tough crystalline structure of cellulose microfibril can be solubilized using ILs to release starch granules stored in cells [108]. Several research studies reported that the usage of ILs is in fact the most energy efficient and least time-consuming method to extract carbohydrate from microalgae biomass in the absence of acid, alkali, and catalyst [109]. Besides, it is reported that the carbohydrate-rich fraction which remains after ILs extraction is suitable to be used as feedstock to produce butanol via fermentation without any further pretreatment [110]. Another study reported the inexpensive choline amino acid-based IL is capable to extract total sugar content of 71 and 21%, respectively, from *C. vulgaris* and *S. platensis* [111].

#### Proteins

Microalgae are one of the protein-rich crops, where their protein yield is said to be comparable to the protein yield of conventional protein sources such as soy, milk, and animal meat. *Spirulina* has been cultivated and marketed in the form of tablets and pills as protein supplements for human consumption [2]. The crude extract of *T. suecica* was reported to contain proteins with emulsification, foaming, and gelation properties which may open up a variety of application options in food industry [112]. Another type of protein that can be extracted from microalgae is R-phycoerythrin, which is a type of phycobiliprotein that is usually used as fluoresce dye in diagnostic and research field [113]. In the study, cholinium-based IL was able to extract 46.5% of R-phycoerythrin from *Gracilaria* sp., which was significantly higher when compared to conventional method [114]. Besides, extraction study of Rubisco, which is an abundant microalgae enzyme, revealed that the IL-based ABS investigated was 3–4 times more efficient in separating complex plant proteins compared to the polyethylene glycol-based extraction [91]. The results have shown the potential of ILs as extractive solvent to separate and purify complex proteins such as enzymes from microalgae for industrial applications. Nevertheless, the functional usage of microalgae proteins extracted using ILs remains largely unexplored at large.

The article "A review on microalgae cultivation and harvesting, and their biomass extraction processing using ionic liquids" was retracted in 2026. Reason: compromised peer review.

#### Bioactive compounds

Although many researches on microalgae have mainly centered around the biofuel production, microalgae metabolites have a variety of functions. Metabolites such as carotenoids are well-known for their antioxidant properties. Examples of such carotenoids which are widely used in pharmaceutical and food industries as nutritive supplements and coloring agents are β-carotene and astaxanthin that are mainly extracted from *D. salina* and *Haematococcus pluvialis*, respectively [115,116]. The use of 1-ethyl-3-methylimidazolium dibutylphosphate for the extraction of astaxanthin from *H. pluvialis* certainly aids the industry in fulfilling the need of the market via vastly improving the extraction yield at a lower energy demand and production cost which in turn makes the product to be more competitive even with the presence of artificially synthesized astaxanthin in the market [117,118]. Other microalgae metabolites of interest include tocopherols, phenolics compounds, flavonoids, and vitamins that have been previously found in microalgae extracts of different species and may be potentially extracted using ILs [119–121]. These compounds have various therapeutics functions such as anti-inflammatory, antimicrobial, anti-viral, antioxidant, and even anticancer effects [122,123].

### Challenges of commercialization of ionic liquids for the extraction of bioproducts from microalgae

Despite the various studies that emphasize on the benefits of ILs for the extraction of microalgae derived bio-compounds, ILs are still to this date not being used commercially. This may be attributed to the toxicity and non-biodegradability of some traditional ILs such as imidazolium-based ILs, which may pose as an environmental risk when they are not properly treated prior to discharge to the environment. In fact, several toxicology studies have reported that conventional ILs are able to disrupt cell membrane and increase reactive oxygen species production in various organisms such as bacteria, fungus, plants, and animal cell lines *in-vitro* and ultimately lead to death. Moreover, due to the complexity of ILs’ molecular structure, they tend to be much harder to be synthesized, and therefore contribute to high production cost and are generally 5–20 times more expensive than conventional solvents. On-going efforts need to be continued to lower down the production cost of ILs, and also optimize their usage.

The article "A review on microalgae cultivation and harvesting, and their biomass extraction processing using ionic liquids" was retracted in 2026. Reason: compromised peer review.

## Conclusions

It is well established that microalgae have tremendous potential as a source of biofuel, food and high value bio-compounds. However, the limitations in productivity of microalgae and the drawbacks of bioprocessing technologies render the fully utilization of microalgae biomass to be impractical. Therefore, more work needs to be done to further improve the existing technology. For instance, more advanced culturing technique should be developed to increase the productivity of microalgae, and novel biotechnology such as gene editing can be attempted to increase the output of bioactive compounds from the microalgae strain. Besides, the ILs studied should be examined for their toxicity before application. In addition, computer simulation can be used to further explore the combination of various cation and anion of ILs to maximize the extraction capacity of desired compounds from microalgae.

## Highlights

- Microalgae cultivation using open ponds (circular and raceway ponds)
- Different designs of photobioreactors: tubular, vertical column, and flat-plate
- Harvesting techniques: filtration, centrifugation, flocculation, and flotation
- Extraction of bioproducts from microalgae using ionic liquid as extractive solvent
- Bioproducts extracted: lipids, carbohydrates, proteins and bioactive compounds
